# Fuzzy Medical Computer Vision Image Restoration and Visual Application

**DOI:** 10.1155/2022/6454550

**Published:** 2022-06-21

**Authors:** Yi Tang, Jin Qiu, Ming Gao

**Affiliations:** ^1^School of Environmental Science and Engineering, Suzhou University of Science and Technology, Suzhou 215009, China; ^2^School of Electronic and Information Engineering, Suzhou University of Science and Technology, Suzhou 215009, China; ^3^School of Mechanical Engineering, Sichuan University, Chengdu 610065, China

## Abstract

In order to shorten the image registration time and improve the imaging quality, this paper proposes a fuzzy medical computer vision image information recovery algorithm based on the fuzzy sparse representation algorithm. Firstly, by constructing a computer vision image acquisition model, the visual feature quantity of the fuzzy medical computer vision image is extracted, and the feature registration design of the fuzzy medical computer vision image is carried out by using the 3D visual reconstruction technology. Then, by establishing a multidimensional histogram structure model, the wavelet multidimensional scale feature detection method is used to achieve grayscale feature extraction of fuzzy medical computer vision images. Finally, the fuzzy sparse representation algorithm is used to automatically optimize the fuzzy medical computer vision images. The experimental results show that the proposed method has a short image information registration time, less than 10 ms, and has a high peak PSNR. When the number of pixels is 700, its peak PSNR can reach 83.5 dB, which is suitable for computer image restoration.

## 1. Introduction

In many discussions, graphics and images are often referred to as “graphic images,” which creates a great deal of ambiguity in the meaning of graphics and images in use. Although they are both represented in numerical form, there is a fundamental difference between storage format and representation. Graphic is an image storage form of the vector structure, which implicitly and uniformly describes the color or brightness of the picture content, and the recorded content is mainly coordinate values or coordinate sequences. An image is an image storage form of a grating structure that divides the image into evenly distributed gratings and explicitly records the photometric value of each pixel. The coordinates of the pixels are implicit in the regular arrangement of their positions. With the development of modern technology, people's requirements for image processing technology are getting higher and higher, and their processing speed and processing accuracy are required to have a high level research. In recent years, people have combined information technology with medicine and used image information processing technology to process medical images to improve the clarity of medical images[1, 2].

In reference [3], a method for segmentation of blurred target edge of brain tumor based on MRI image is proposed to improve the accuracy of image segmentation and obtain clearer images. The method first uses the ink sampling method to select the image, completes the image denoising and grayscale processing according to the PM model and the maximum-minimum value method, and then extracts the pixel point features of the processed image according to the sliding window and constructs the image mixture model. And finally, the EM algorithm is used to complete the solution of the blurred target edge of the image, realize image segmentation, and improve the clarity of the acquired image. Although this method can optimize the image to a certain extent, it is time-consuming and the feature parsing ability is not ideal. In reference [4], a fuzzy image recognition method based on LoG edge detection and enhanced local phase quantization is proposed. Value quantization to obtain phase features that can accurately describe the frequency domain of the image and use the multiscale LoG operator to extract the edge features of the image to highlight the key details of the image. The phase feature histogram was obtained in the frequency domain, and the edge feature was obtained in the space domain. The combination of histograms improves the algorithm's recognition performance and robustness to blur, which can improve image sharpness, but this method is limited by poor adaptability and low output pixel intensity. Many image processing techniques work at the local, single-pixel level. One of the fundamental problems with such algorithms is scale. For example, the edge corresponds to the gradient of the image function, and the edge detection is calculated according to the difference between the pixels in a neighboring city. Similarly, the sensitivity of shape descriptors to scale (image resolution) is an unwelcome feature of most such descriptors. This allows the shape description to vary with the scale, resulting in different results at different resolutions. Therefore, the selection of neighborhood scale becomes one of the main problems faced by many algorithms, because the selection of appropriate scale often depends on the size of the object to be investigated, which is often unknown in the initial stage of image processing. Although the accurate scale estimation cannot be obtained at the beginning of image processing, the approximate pixel resolution expression and the general scale description are very useful for choosing the appropriate processing method in some applications.

Aiming at above problems, a fuzzy medical computer vision image information recovery algorithm based on fuzzy sparse representation algorithm is proposed in this study. The computer vision image acquisition model and the multidimensional histogram structure model of the fuzzy medical computer vision image are constructed [5]. The wavelet multidimensional scale feature detection method is used to extract the gray scale feature and realize the restoration of the fuzzy medical computer vision image. The simulation experiment shows that the proposed method can improve the restoration of the fuzzy medical computer vision image.

## 2. Computer Vision Image Acquisition and Information Enhancement Processing

### 2.1. Computer Vision Image Acquisition Model

Resolution refers to the spatial fine degree of image digitalization. There are two kinds of resolution: display resolution and image resolution. The essence of image resolution is to divide the pixel density of the image when digitizing the image, namely, the number of pixels per unit length. The display resolution is the number of pixels that a word image can display on an output device (such as a display screen or printer) and the dot space between the pixels displayed. The image resolution indicates the actual precision of the digital image, and the display resolution indicates the precision of the digital image. Digital images with different image resolutions have the same display resolution on the same output device.

To realize the optimal design of information restoration of fuzzy medical computer vision image, firstly, the 3D vision information acquisition model is constructed, and the computer vision image acquisition is conducted by combining the method of feature registration [6–8]. The spatial visual feature reconstruction of fuzzy medical computer vision image is realized by using multidimensional 3D tracking and information sampling party, and the point scanning and tracking technology is combined with the method of feature registration. The three-dimensional vision sampling image of fuzzy medical computer vision image space is obtained by using the method of image combination sampling in *s*(*X*, *Y*). The distributed information sampling output of fuzzy medical computer vision image is obtained as follows:

(1) $$\begin{array}{c} N\text{cut}\left(A,B\right)=\frac{\text{cut}\left(A,B\right)}{\text{assoc}\left(A,V\right)}+\frac{\text{cut}\left(A,B\right)}{\text{assoc}\left(B,V\right)}, \end{array}$$

wherein, assoc(*A*, *V*) represents the pixel subset of fuzzy medical computer vision image under machine vision. By using the template feature matching method, the collected fuzzy medical computer vision image is reconstructed, and their outputs are obtained.

(2) $$\begin{array}{c} W_{u}u\left(a,b_{m}\right)=\frac{1}{\sqrt{a}}\int_{-aT/2+b_{m}}^{T/2}{\left|\frac{1}{\sqrt{T}}\right|}^{2}dt=\frac{1}{\sqrt{a}T}\left(\frac{T}{2}+\frac{aT}{2}-b_{m}\right). \end{array}$$

In the pixel distribution space, the gray scale of fuzzy medical computer vision image is calculated, and its multilayer segmentation model is constructed, which is expressed by

(3) $$\begin{array}{c} d_{i+1}=2F\left(x_{i+1}+\frac{1}{2},y_{i}+2\right)=\left\{\begin{array}{cc} 2\left[\Delta x\left(y_{i}+2\right)-\Delta y\left(x_{i,r}+\frac{1}{2}-\Delta xB\right)\right], & d_{i}\leq 0,\\ 2\left[\Delta x\left(y_{i}+2\right)-\Delta y\left(x_{i,r}+1+\frac{1}{2}-\Delta xB\right)\right], & d_{i}>0. \end{array}\right. \end{array}$$

In the fuzzy region, CT imaging technology is used for image acquisition, and the output of computer vision image acquisition is obtained:

(4) $$\begin{array}{c} P\left(y_{w_{3}}\left|x_{w_{3}}\right.,\theta ,\beta \right)\propto P\left(y_{w_{3}}\left|x_{w_{3}}\right.,\theta \right)\left(y_{w_{3}}\left|\beta_{i}\right.\right)\propto \overset{K}{\underset{k=1}{\prod }}\alpha_{k}\frac{1}{\sqrt{2{\pi \sigma }_{k}^{2}}}\exp\left\{-\frac{{\left(x_{i}-\mu_{k}\right)}^{2}}{2\sigma_{k}^{2}}\right\}\cdot \frac{1}{Z\left(\beta_{i}\right)}\exp\left(-\underset{c\subset C}{\sum }V_{c}\left(Y,\beta_{i}\right)\right)\propto \overset{K}{\underset{k=1}{\prod }}\frac{\alpha_{k}}{Z\left(\beta_{i}\right)\sqrt{2{\pi \sigma }_{k}^{2}}}\cdot \exp\left\{-\left[\overset{K}{\underset{k=1}{\sum }}\frac{{\left(x_{i}-\mu_{k}\right)}^{2}}{2\sigma_{k}^{2}}+\underset{c\subset C}{\sum }V_{c}\left(Y,\beta_{i}\right)\right]\right\}. \end{array}$$

Each template in the visual image visual space of the fuzzy medical compute is subjected to grid segmentation, and the local association frame binary reconstruction is performed in the *m*∗*n* area, and a fuzzy information reconstruction model of the fuzzy medical computer vision image is constructed, so that the regional characteristic distribution point of the blurred medical computer vision image is obtained:

(5) $$\begin{array}{c} J\left(x\right)=\frac{I\left(x\right)-A}{\max\left(t\left(x\right),t_{0}\right)}+A, \end{array}$$

wherein, *t*_0_ denotes the structural similarity of the fuzzy medical computer vision image, the template matching is carried out in the image 3∗3 neighborhood structure, and the spatial segmentation and information enhancement processing are conducted [9, 10].

### 2.2. Image Information Enhancement

The image processing method is used to obtain images of scenes with high dynamic brightness range, which can fully show the rich details of light and dark areas in complex lighting scenes. The method of high dynamic range image synthesis based on multiexposure image sequence is one of the common methods of high dynamic range image synthesis. At present, Debevec algorithm, as an accurate and stable camera response function calibration algorithm, has been adopted by many high dynamic range image processing software. However, Debevec algorithm has some shortcomings, such as low camera response function calibration efficiency and lack of effective denoising processing, resulting in poor synthesis of high dynamic range images.

After dividing the long line into several small local regions, each local region has the property of a straight line. The larger local area connected by small local areas still has this linear property. Therefore, a longer line segment can be constructed gradually by connecting local line edges. Based on this idea, a hierarchical structured line extraction algorithm is put forward, which can be expanded as follows:

- Image edge support area detection and edge refinement

According to the isotropic circular window structure. In accordance with the principle of linearity and adjacency, the adjacent underlying structures are connected to form a higher structure region.

- Repeat steps until no regions exist that can be combined

(4) The linear regression method is used to extract line parameters from each set of regions obtained by step (3). When extracting the line parameters, the supporting region is divided into several subregions and the dominant points are extracted in each subregion. The line parameters are obtained by fitting the dominant points of each subregion.

- Connect short straight segments according to the principles of similarity and proximity

The feature registration design of fuzzy medical computer vision image is conducted by using 3D vision reconstruction technology. The vector set of visual feature distribution of fuzzy medical computer vision image is calculated [11–13]. The quantitative feature distribution set of fuzzy medical computer vision image region segmentation is obtained:

(6) $$\begin{array}{c} w\left(i,j\right)=\frac{1}{Z\left(i\right)}\exp\left(-\frac{d\left(i,j\right)}{h^{2}}\right), \end{array}$$

where *Z*(*i*) = ∑_*j*∈*Ω*_exp(−*d*(*i*, *j*)/*h*^2^) is the spatial visual gradient feature of fuzzy medical computer vision image, the visual feature quantity of fuzzy medical computer vision image is extracted, the feature registration design of fuzzy medical computer vision image is conducted, the gradient model sign of fuzzy medical computer vision image is defined, the spatial visual feature registration of fuzzy medical computer vision image is carried out by unit moving scale association allocation method, the gradient model feature is extracted, the fuzzy region is processed by block fusion, and the gradient model reconstruction and information fusion operator is used to detect the edge of fuzzy medical computer vision image.

(7) $$\begin{array}{c} \underset{c}{\min}\left(\underset{y\in \Omega \left(x\right)}{\min}\left(\frac{I^{c}\left(y\right)}{A^{c}}\right)\right)=\tilde{t}\left(x\right)\underset{c}{\min}\left(\underset{y\in \Omega \left(x\right)}{\min}\left(\frac{J^{c}\left(y\right)}{A^{c}}\right)\right)+\left(1-\tilde{t}\left(x\right)\right), \end{array}$$

where $\tilde{t}\left(x\right)$ represents the matching set of image frame feature points, *A*^*c*^ represents the statistical feature of spatial pixels of fuzzy medical computer vision image, and *I*^*c*^(*y*) represents the edge information intensity value of the first feature sampling point of image. The feature points of fuzzy medical computer vision image are obtained as follows:

(8) $$\begin{array}{c} {\text{bnr}}_{\beta }\left(X\right)=R_{\beta }X-R_{\beta }X_{1}. \end{array}$$

By establishing the high-precision feature registration model of fuzzy medical computer vision image, the spatial vision distribution pixel value of image is obtained:

(9) $$\begin{array}{c} w\left(d_{ij}\right)=f\left(\left|x_{i}-x_{j}\right|\right)=\frac{1}{\sqrt{2\pi }}\exp\left\{\frac{{\left(x_{i}-x_{j}\right)}^{2}}{2}\right\}. \end{array}$$

The similarity feature resolution model of fuzzy medical computer vision image is established to conduct the spatial vision reconstruction of image [14, 15]. In the regional pixel distribution interval, the scene coordinate is *M* × *N*. The segmented region feature registration of fuzzy medical computer vision image is carried out, and the feature points are added to the reconstructed scene to realize the visual feature extraction and information enhancement, and the output pixel value is

(10) $$\begin{array}{c} \beta_{i}=\exp\left\{-\frac{{\left|x_{i}-x_{j}\right|}^{2}}{2\sigma^{2}}\right\}\frac{1}{\text{dist}\left(x_{i},x_{j}\right)}. \end{array}$$

In this paper, the multilayer mesh region distribution model of the fuzzy medical computer vision image is constructed, and the image information enhancement processing is conducted [16–18].

## 3. Optimization of Image Information Recovery Algorithm for Fuzzy Medical Computer

### 3.1. Fuzzy Medical Computer Vision Image Visual Feature Extraction

Computer image analysis usually refers to the process of finding out which object is contained in the image by computer. Point feature, line feature, edge feature, and region feature are basic data for image matching and 3D reconstruction. In the image, the edge is the boundary between the target connected region and other regions. The edge feature corresponds to the part of the image where the brightness changes. In computer vision, there are edge enhancement and edge detection. Image edge detection is the key to deal with many visual problems. The extraction and expression of feature points provide effective support for multiview correspondence of stereo vision. Feature-based stereo matching algorithm needs edge feature, region feature, and point feature as input. In addition, feature extraction and expression are a necessary step for image understanding. Although only a correct understanding of the image can obtain good feature extraction, the extraction of basic features is the first step to solve the problem.

Here, we study it from two aspects: one is to use the simulated image for experiment, and the other is to use the real foggy image for research. Finally, we compare the problems in the two aspects:

1. First aspect

- The first step of the program is to simulate the processing of foggy image, assign a value to the color a of atmospheric light, and assign a value to multiple *R*
- The second step is to generate the original fog free image with multiple albedo values
- The third step is to add fog to the original image
- The fourth step is to output the fog free image calculated by the proposed algorithm
- The fifth step is to compare the restored image with the original non fog image (compare *T*, *L* values)

(2) Second aspect

- In the first step of real fog image processing, assign a value to the color a of atmospheric light and set the window size
- The second step is to input the foggy image
- The third step is to output the fogless image

The computer vision image acquisition model is used for constructing the visual image feature registration of the fuzzy medical computer, and information enhancement of the blurred medical computer vision image is implemented using the high-resolution visual information enhancement technology [19]. A fuzzy medical computer vision image information recovery algorithm based on fuzzy sparse representation algorithm is presented in this paper. In that method, the visual characteristic amount of the visual image of the fuzzy medical compute is extracted, a 3D visual reconstruction technique is employed for the image feature registration design of the fuzzy medical computer vision image, and the visual image space visual reconstruction of the fuzzy medical computer is conducted using template matching method. The multifractal technology is used for the block matching of the visual feature of the visual image of the fuzzy medical computer, the detail information of different resolutions is matched with the characteristic matching, and the multilevel multidirection decomposition method is adopted for obtaining the similar characteristic quantity of the visual image space of the fuzzy medical computer:

(11) $$\begin{array}{c} s\left(k\right)=\phi \cdot s\left(k-1\right)+w\left(k\right), \end{array}$$

where

(12) $$\begin{array}{c} \phi =\left(\begin{array}{ccccc} 1 & 0 & 0 & 0 & 0\\ 0 & 1 & 1 & 0 & 0\\ 0 & 0 & 1 & 0 & 0\\ 0 & 0 & 0 & 1 & 1\\ 0 & 0 & 0 & 0 & 1 \end{array}\right),\\ w\left(k\right)=\left(\begin{array}{c} N\left(0,\sigma_{\theta \left(k\right)}\right)\\ 0\\ N\left(0,\sigma_{x\left(k\right)}\right)\\ 0\\ N\left(0,\sigma_{y\left(k\right)}\right) \end{array}\right). \end{array}$$

The spatial vision feature distribution value of fuzzy medical computer vision image is extracted, and the *R*, *G*, and *B* components of fuzzy medical computer vision image are obtained by the RGB decomposition method. Based on Gaussian mixture model, the feature extraction output of fuzzy medical computer vision image is obtained in feature template *m* ≤ *n*.

(13) $$\begin{array}{c} E\left[f\left(\theta ,k\right)\right]=0,\forall \theta \in \left[-\pi ,\pi \right],\forall k\in Z. \end{array}$$

The adaptive fusion and optimal segmentation of fuzzy medical computer vision image are conducted [20–25]. Based on the feature segmentation results, the multilayer spatial structure feature registration and fusion clustering of image are implemented, and the information enhancement and visual information feature extraction of fuzzy medical computer vision image are realized as:

(14) $$\begin{array}{c} s\left(k\right)=\phi \cdot s\left(k-1\right)+w\left(k\right), \end{array}$$

(15) $$\begin{array}{c} T_{i,j}\left(t\right)=\frac{\left|p_{i,j}\left(t\right)-\Delta p\left(t\right)\right|}{p_{i,j}\left(t\right)}, \end{array}$$

(16) $$\begin{array}{c} U_{i,j}\left(t\right)=\exp\left[-b{\left[z_{i}\left(t\right)-z_{j}\left(t\right)\right]}^{2}\right], \end{array}$$

where *p*_*i*,*j*_(*t*) represents the displacement characteristic of fuzzy medical computer vision image at *T* time, *sp*_*i*,*j*_(*t*) represents the exchange fitting function, Δ*p*(*t*) represents the reference value of standard image, and *z*_*i*_(*t*) represents the feature output of similarity image. The visual feature quantity of fuzzy medical computer vision image is extracted, based on which the machine learning and optimization are conducted [26–32]. The schematic diagram of extraction results is shown in Figure 1.

The feature points identified by the above methods have some feature discernibility. In some applications, it is of great importance to not only obtain positioning characteristics of interest points but also other features to distinguish them from other interest points. If every point feature on the image has a unique distinctive feature label, it is undoubtedly beneficial to the application of point feature. However, the two demands are contradictory. To obtain an accurate location, it needs to use a small window, while to increase the distinction, it is necessary to increase the window. It is not necessary to distinguish every feature point completely. As long as a certain method can be used to divide the point features of an image into more classes will be greatly convenient for application. One way to obtain highly discriminative features is to increase the discernibility of features by using a wide range of information. For example, feature vectors can be constructed using color and brightness changes in the image in the window adjacent to the point of interest, or geometric features can be used. The specific method of constructing the point eigenvector depends on the specific purpose of application. For example, for stereo image matching, scale invariant feature vectors and rotation invariant feature vectors based on geometric features can be constructed. For wide baseline stereo matching, affine invariant feature vectors should be constructed to deal with the large projection deformation.

### 3.2. Machine Learning Optimization

Space vision rotation and feature extraction of fuzzy medical computer vision image is conducted in a 4-to-4 subblock segmentation model. A block feature matching method is adopted, the original fuzzy medical computer vision image is correlated frame sampling, the quantization characteristic coding method is adopted, the coding design of the fuzzy medical computer vision image is conducted in the *D*-dimensional space, the fuzzy sparse representation algorithm is employed to perform the self-adaptive registration and optimization of the blurred medical computer vision image, and the registration output is

(17) $$\begin{array}{c} u\left(x,y;t\right)=G\left(x,y;t\right), \end{array}$$

wherein Δ*u* is the local correlation pixel, *σ* is the horizontal difference characteristic quantity of the fuzzy medical computer vision image, in the *A*_*g*_ region, the adaptive machine learning optimization model of the brain function time series diagram is obtained, the corner point detection of the fuzzy medical computer vision image is conducted in the gradient direction, and the information recovery is performed by using the wavelet multidimensional scale feature detection method.

(18) $$\begin{array}{c} \left\{\begin{array}{cc} x=R\sin\eta \cos\phi , & 0\leq \phi \leq 2\pi ,\\ y=R\sin\eta \sin\phi , & 0\leq \eta \leq \pi ,\\ z=R\cos\eta , & \;R=\frac{D}{2}, \end{array}\right. \end{array}$$

where *η* denotes the edge brightness of the line fuzzy medical computer vision image, *ϕ* denotes the sparse feature component, *R* denotes the template matching coefficient, and *D* denotes the edge fuzzy pixel set. Based on the above analysis, the wavelet multidimensional scale feature detection method is adopted for grayscale feature extraction of fuzzy medical computer vision image, and the fuzzy sparse representation algorithm is employed to optimize the information recovery of fuzzy image, so as to improve the registration accuracy [20–24, 33–39]. The matching diagram is shown in Figure 2.

## 4. Simulation

The experiments in this paper are carried out on a laptop with Windows 10 operating system and 8 GB memory. The model is constructed using MATLAB simulation software to verify the feasibility of the proposed method. Before using MATLAB to process images, you need to read the images in different formats and then convert them into several types supported by MATLAB. After reading the image, you need to convert the image type before processing. It is to solve these problems, through which it can complete the interaction with other programming environments, take what they need, give full play to the strengths of MATLAB numerical calculation, and avoid the shortcomings of MATLAB execution efficiency. The pixel set of the fuzzy medical computer vision image is 150 × 150, and each fuzzy medical computer vision image is randomly sampled with 100 pixels. According to the above simulation parameters, the fuzzy medical computer vision image registration is performed, and the original image is shown in Figure 3.

Taking the image of Figure 4 as the input, the fuzzy medical computer vision image vision feature quantity is extracted. The fuzzy medical computer vision image feature registration design is conducted by using the 3D vision reconstruction technology, as shown in Figure 5.

The time consumption in image registration by different methods is tested, as shown in Table 1.

Table 2 shows that the proposed method can improve the PSNR of image registration and enhance the imaging quality.

## 5. Conclusions

In order to improve the registration efficiency and registration accuracy in medical image processing, this paper proposes a fuzzy medical computer vision image information recovery algorithm based on the fuzzy sparse representation algorithm. The computer vision image acquisition model is used to extract the visual features of the fuzzy medical computer vision image. 3D visual reconstruction technology is used for image registration. The multidimensional histogram structure model of the visual image is established, and the grayscale feature of the blurred image is extracted by the wavelet multidimensional scale feature detection method. Based on the feature extraction results, a fuzzy sparse representation algorithm is used to automatically optimize the restoration of medical computer vision image information. Simulation experiments are used to prove the effectiveness of this method. Compared with the comparison method, the registration time of this method is less than 10 ms, and the PSNR peak of its image registration reaches 83.5, which is better than the comparison method, which proves that this method can improve the fuzzy medical computer. Peak signal-to-noise ratio and registration accuracy of visual image registration to obtain clearer medical images. Although the method in this paper has certain research results, the existing algorithm is not very effective in some cases due to the large amount of calculation. There are still many problems to be improved and solved. In the future, it is necessary to combine advanced technology to develop commercial. Image synthesis and visualization algorithms with good real-time performance and high dynamic range improve the registration efficiency and registration accuracy of image processing.

## Figures and Tables

**Figure 1:** Example of extraction results.

**Figure 2:** Matches the results.

**Figure 3:** Original blurred medical computer vision image.

**Figure 4:** Feature point extraction to achieve defogging effect diagram.

**Figure 5:** Visual image registration output of the fuzzy medical computer.

**Table 1:** Time-cost comparison of image information recovery (unit: ms).

Image pixel	Proposed method	Method in reference [4]	Method in reference [5]
100	2.57	16.72	15.37
300	5.64	32.57	24.71
500	7.68	35.75	34.18
700	8.76	62.75	48.59

**Table 2:** Comparison of peak PSNR (unit: dB)).

Image pixel	Proposed method	Method in reference [4]	Method in reference [5]
100	46.4	31.5	25.1
300	65.3	37.4	36.4
500	72.5	45.9	38.2
700	83.5	47.8	44.7

## Data Availability

The data used to support the findings of this study are available from the corresponding author upon request.
